# Research on Association between Levels of Serum Adiponectin, Hs-CRP, and sICAM-1 and Hypertensive Cerebrovascular Complications

This article has been retracted.

**DOI:** 10.1155/2021/4455038

**Published:** 2021-09-13

**Authors:** Haijun Niu, Rongyan Jiang, Songwu Dong, Linhu Xia, Hongyi Fang

**Affiliations:** Department of Cardiology, Bozhou People's Hospital, Bozhou, 236800 Anhui Province, China

## Abstract

The study is aimed at studying the association between the levels of serum adiponectin (ADPN), high-sensitivity C-reactive protein (hs-CRP), and soluble intercellular adhesion molecule-1 (sICAM-1) and hypertensive cerebrovascular complications. 50 patients with hypertensive cerebrovascular disease treated in Gansu Provincial Hospital from December 2016 to December 2018 were selected as the experimental group, and 50 normal people who underwent physical examination were selected as the control group. The blood pressure, heart rate, and the complications were recorded, and the serum blood lipid indexes were detected. Moreover, the content of serum ADPN, hs-CRP, and sICAM-1; the neurological indexes; brain-derived neurotrophic factor (BNDF); and neurone-specific enolase (NSE) were also determined using ELISA. The content of aspartate aminotransferase (AST), alanine aminotransferase (ALT), blood urea nitrogen (BUN), and serum creatinine (SCR) in the experimental group was significantly higher than that in control group (*p* < 0.05); the incidence of cerebrovascular complications, systolic blood pressure, diastolic blood pressure, and heart rate increased (*p* < 0.05); the content of total cholesterol (TC), triglyceride (TG), low-density lipoprotein (LDL), high-density lipoprotein (HDL), hs-CRP, and sICAM-1 obviously rose (*p* < 0.05); and the content of ADPN and HDL obviously declined (*p* < 0.05). Besides, the experimental group had evidently lower systolic blood flow velocity (Vs), diastolic blood flow velocity (Vd), and mean blood flow velocity (Vm) and evidently higher pulsatility index (PI) (*p* < 0.05). The levels of S100 and NSE in the experimental group increased significantly, and the level of BNDF decreased significantly (*p* < 0.05). In patients with hypertensive cerebrovascular disease, the level of ADPN declines; the levels of hs-CRP and sICAM-1 rise; the incidence rate of cerebrovascular complications is elevated; and there are changes in the blood lipid, cerebrovascular hemodynamic, and neurological indexes, thereby further promoting the occurrence and development of hypertensive cerebrovascular disease.

## 1. Introduction

Cardiovascular disease has become an important cause of death and disability with age. The deaths caused by cardiovascular disease account for more than 20% in the elderly in Western Europe and North America. Cardiovascular disease may be a more horrible disease than death for the elderly. Hypertension is a major risk factor for stroke, and the incidence rate of atherosclerosis cerebral infarction in patients with hypertension is about 4 times than that in patients with normal blood pressure [1]. The correlation between the increased incidence of stroke and the increased arterial pressure in the elderly has been confirmed [2]. According to experimental and clinical evidence, the cerebrovascular system is highly sensitive to arterial hypertension. The development of cerebrovascular and brain parenchymal changes in patients with chronic hypertension has also been documented [3]. Chronic hypertension leads to cerebrovascular morphological changes, increases the risk of cerebral hypoperfusion, reduces oxygen supply to brain tissues, and raises the likelihood of ischemia [4]. The main role of hypertension in stroke and other cerebrovascular diseases has been fully confirmed. Most studies focus on the arterial vessel system, but there is less information about the cerebrovascular changes caused by hypertension [5]. Recent evidence suggests that hypertension is the most important risk factor for brain compartment syndrome and cerebral hemorrhage compared with other forms of stroke, indicating the role of cerebral arterial changes due to hypertension in the pathogenesis. In the previous small-scale analysis of the PIUMA study, it was found that elevated blood pressure has a univariate association with the cardiocerebrovascular and peripheral vascular events [6]. Therefore, analyzing the cerebral arterial changes related to hypertension is helpful to better understand the pathophysiology of hypertensive cerebral injury. Currently, the impact of hypertension on the prognosis of cardiocerebrovascular diseases remains unclear, so further research is needed.

Adiponectin (ADPN) is a kind of recently discovered adipocytokine produced and secreted by adipose tissues [7]. Studies have shown that there is a significant negative correlation between plasma ADPN and insulin resistance [8], while a higher level of ADPN is associated with a lower incidence of type 2 diabetes mellitus according to prospective studies [9]. ADPN has an anti-inflammatory effect, and it also has a negative correlation with C-reactive protein (CRP) and other inflammatory markers [10]. The level of ADPN declines in subjects with subclinical atherosclerosis markers and patients with clinical manifestations of coronary heart disease [11, 12]. High-sensitivity CRP (hs-CRP), an acute-phase protein associated with systemic inflammation, has been proven to increase in patients with coronary heart disease [13, 14], but whether its content rises in patients with cerebrovascular disease needs further studies. Soluble intercellular adhesion molecule-1 (sICAM-1) has little or no expression in normal blood vessels. It can participate in inflammation and adhesion reactions, leading to vasoconstriction, ultimately resulting in vascular restenosis and cardiovascular events [15]. The treatment of cardiovascular disease can not only effectively prevent platelet cross-linking and aggregation, but also inhibit the expressions of inflammatory factors, chemokines, and adhesion factors, thereby reducing the level of sICAM-1, improving the prognosis of patients, lowering the incidence of adverse cardiovascular events, and enhancing the quality of life of patients [16]. However, there are few studies on the effects of the above three factors on hypertensive cerebrovascular complications, so their influences on hypertensive cerebrovascular complications were further explored in the present study.

In the present study, patients with hypertensive cerebrovascular disease and normal people receiving physical examination were collected as experimental subjects. Then, venous blood was drawn to detect the serum routine biochemical indexes of hepatic and renal function, blood pressure and heart rate were measured in each group, and blood lipid indexes were detected. Moreover, the content of serum ADPN, hs-CRP, and sICAM-1 was determined using enzyme-linked immunosorbent assay (ELISA); the hemodynamic indexes were detected; and the neurological indexes of serum brain-derived neurotrophic factor (BNDF) and neurone-specific enolase (NSE) were also determined using ELISA, hoping to provide theoretical and experimental basis for the prevention and treatment of hypertensive cerebrovascular disease.

## 2. Clinical Data and Experimental Methods

### 2.1. General Data

A total of 50 patients with hypertensive cerebrovascular disease treated in Gansu Provincial Hospital from December 2016 to December 2018 were selected as the experimental group. In addition, 50 people with normal physical examination were selected as the control group, and they all signed the informed consent form. Inclusion criteria are as follows: subjects meeting the diagnostic criteria for hypertension in the Hypertension Prevention and Treatment Guideline, those who volunteered to participate in the study and signed the informed consent, and those receiving no treatment previously. Exclusion criteria are as follows: diabetic patients, those with secondary infection + severe hepatic and renal dysfunction, or those with acute myocardial infarction. All clinical specimens in this experiment were obtained upon the agreement of the Ethics Committee of Gansu Provincial Hospital and family members. The clinical research protocol was approved by the Ethics Committee of Gansu Provincial Hospital. The specific clinical data of the patients were collected at the time of admission, including age, gender, weight, physical condition, and hypertension classification (Table 1), and there was no significant difference.

### 2.2. Detection of Serum Blood Urea Nitrogen (BUN), Serum Creatinine (SCR), Aspartate Aminotransferase (AST), and Alanine Aminotransferase (ALT)

Serum biochemical indexes of hepatic and renal function will be affected by many diseases, and hypertensive cerebrovascular disease is no exception. Five mL of venous blood was drawn from the arm and placed in an EP tube containing an anticoagulant, followed by centrifugation at 2000 g for 15 min at room temperature. The supernatant was collected to detect the hepatic and renal function indexes BUN, SCR, AST, and ALT, so as to provide an important theoretical reference for early treatment.

### 2.3. Detection of Blood Pressure and Heart Rate and Recording of Complications

The left ventricles of patients were auscultated using a stethoscope in a quiet state, and the heartbeats per minute were recorded 3 times. After the cuff of the sphygmomanometer was wrapped around the patient's arm, the rubber ball was squeezed to gradually elevate the mercury column until no pulse of the brachial artery was heard by the stethoscope, at which moment the value in the sphygmomanometer was the systolic blood pressure. Then, the cuff was slowly deflated, and the value in the sphygmomanometer was the diastolic blood pressure at the moment when the sound turned from strong to weak. In the experimental group, the patients were grouped based on the expressions of serum ADPN, hs-CRP, and sICAM-1, and the cerebrovascular complications were recorded, mainly including cerebral hemorrhage, stroke, and cerebral infarction. The specific diagnostic criteria are as follows: a history of hypertension, heart disease, etc.; acute onset of all or local brain damage; and corresponding lesions or related diseases detected by CT. In the experimental group, ADPN < 2 mg/L, hs − CRP < 4 mg/L, and sICAM − 1 < 500 ng/mL indicated the low expression, otherwise the high expression [17–19].

### 2.4. Detection of Blood Lipid Indexes: Total Cholesterol (TC), Triglyceride (TG), Low-Density Lipoprotein (LDL), and High-Density Lipoprotein (HDL)

In patients with hypertension, the biochemical indexes of blood lipids will be changed, so their changes can be detected to indicate the occurrence and development of disease. Five mL of fasting peripheral venous blood was drawn in the morning and placed in the EP tube containing anticoagulant EDTA, followed by centrifugation at 3500 g for 10 min at room temperature. The supernatant was collected to detect the blood lipid indexes TG, TC, LDL, and HDL, so as to provide an important theoretical reference for early treatment.

### 2.5. Detection of Content of ADPN, Hs-CRP, and sICAM-1 via ELISA and Analysis of Correlation with Incidence Rate of Cerebrovascular Complications

In the morning, 5 mL of peripheral venous blood was drawn on an empty stomach in each group, placed in an EP tube containing anticoagulant EDTA, and centrifuged at 3000 g for 10 min at room temperature. The supernatant was collected to detect the changes in content of serum ADPN, hs-CRP, and sICAM-1 according to the instructions of the ELISA kits (Nanjing Jiancheng Bioengineering Institute). Then, the absorbance of indexes in each group was measured using a microplate reader. The correlation of ADPN, hs-CRP, and sICAM-1 with the incidence rate of cerebrovascular complications was analyzed using the Pearson method.

### 2.6. Cerebrovascular Hemodynamic Detection

The systolic blood flow velocity (Vs), diastolic blood flow velocity (Vd), mean blood flow velocity (Vm), and pulsatility index (PI) of each blood vessel were observed and recorded using the MEDENG CBA CV-300 cerebrovascular hemodynamic analyzer (probe frequency: 2 MHz) according to the manufacturer's instructions.

### 2.7. Detection of Serum Neurological Indexes through ELISA

In each group, 5 mL of fasting peripheral venous blood was drawn in the morning and placed in the EP tube containing anticoagulant EDTA, followed by centrifugation at 3000 g for 10 min at room temperature. The supernatant was collected according to the instructions of the ELISA kit (Nanjing Jiancheng Bioengineering Institute), and changes of serum S100, NSE, and BNDF were detected. Then, the absorbance of indexes in each group was measured using the microplate reader.

### 2.8. Statistical Analysis

All raw data obtained in the experiments were statistically analyzed using SPSS 21.0 software, and multiple comparisons were performed. The experimental results were expressed as mean ± standard deviation ($\bar{\chi }\pm \text{SD}$). Correlation analysis was performed using the Pearson method. *p* < 0.05 suggested that the difference was statistically significant. The bar graph was plotted using GraphPad Prism 5.0.

## 3. Results

### 3.1. Serum Hepatic and Renal Function Indexes

As shown in Table 2, the content of AST, ALT, SCR, and BUN in the experimental group was significantly increased (*p* < 0.05), indicating the changes in liver and kidney metabolic functions in patients with hypertensive cerebrovascular disease, which can provide a basis for early prediction of disease.

### 3.2. Blood Pressure and Heart Rate

As shown in Table 3, the systolic and diastolic blood pressure and heart rate were all obviously increased in the experimental group compared with those in the control group (*p* < 0.05), suggesting the significant changes in blood pressure and heart rate of patients with hypertensive cerebrovascular disease.

### 3.3. Blood Lipid Indexes

The blood lipid index level will change when there is hypertension, so the blood lipid indexes TG, TC, LDL, and HDL are measured. The results showed that in the experimental group, the content of TC, TG, and LDL obviously rose (*p* < 0.05), while the content of HDL obviously declined compared with those in the control group (*p* < 0.05) (Figure 1), suggesting hyperlipidemia in patients with hypertensive cerebrovascular disease.

### 3.4. Levels of Serum ADPN, Hs-CRP, and sICAM-1 Detected Using ELISA

In the experimental group, the content of ADPN was evidently decreased (*p* < 0.05), while that of hs-CRP and sICAM-1 was evidently increased (Table 4).

### 3.5. Content of Serum S100, NSE, and BNDF Detected Using ELISA

In the experimental group, the levels of S100 and NSE were significantly increased (*p* < 0.05), while the BNDF level was significantly decreased (*p* < 0.05) (Table 5).

### 3.6. Cerebrovascular Complications in the Experimental Group

In the experimental group, the patients were grouped based on the expressions of serum ADPN, hs-CRP, and sICAM-1, and the cerebrovascular complications were recorded. As shown in Table 6, there were 14 postoperative complications in the experimental group, and the incidence of cerebrovascular complications was 28%.

### 3.7. Cerebrovascular Hemodynamic Detection Results

The experimental group had evidently lower Vs, Vd, and Vm (*p* < 0.05) and evidently higher PI (*p* < 0.05) (Table 7).

### 3.8. Correlation of Serum ADPN, Hs-CRP, and sICAM-1 Levels with Incidence Rate of Hypertensive Cerebrovascular Complications

In the experimental group, ADPN was negatively correlated with the incidence rate of cerebrovascular complications (*p* < 0.05), while hs-CRP and sICAM-1 were positively correlated with the incidence rate of cerebrovascular complications (*p* < 0.05) (Table 8).

## 4. Discussion

Hypertension is the most important risk factor for cerebral hemorrhage and cerebral infarction, as well as a major risk factor for cerebral hemorrhage. More than 75% of patients with hypertension and more than 80% of patients with cerebral hemorrhage are aged 50-70 years old. Cerebrovascular changes in hypertension, mainly including the increase in the arterial wall thickness, accompanied by the increased media/lumen ratio [20], are closely related to the degree of hypertension. Lumen changes in the cerebrovascular system occur less frequently than those in other vascular beds. Hypertensive cerebral circulation has been extensively analyzed in the widely used hypertensive animal models [21]. The above studies suggest that some structural changes of cerebral arteries in spontaneously hypertensive rats are related to the occurrence and development of hypertension. A higher media/lumen ratio is one of the major changes found in the cerebral arteries of hypertensive animals. It is believed that in hypertensive patients, media thickening accompanied by lumen stenosis are important changes [22, 23]. In this study, the contents of AST, ALT, SCR, and BUN in the experimental group were significantly increased, indicating that the liver and kidney metabolic functions of patients with hypertensive cerebrovascular disease have changed, which can provide a basis for early prediction of disease. The systolic and diastolic blood pressure and heart rate were all obviously increased in the experimental group compared with those in the control group, suggesting the significant changes in blood pressure and heart rate of patients with hypertensive cerebrovascular disease. Studies have demonstrated that the clinical benefits of drug therapy for cerebrovascular complications are mainly attributed to its ability to reduce the levels of blood lipid indexes TC, TG, and LDL [24]. In this study, the blood lipid indexes TG, TC, LDL, and HDL were determined. The results showed that in the experimental group, the content of TC, TG, and LDL obviously rose, while the content of HDL obviously declined compared with those in the control group, suggesting hyperlipidemia in patients with hypertensive cerebrovascular disease. These changes indicate that hypertensive cerebrovascular complications will induce a series of reactions; significantly change liver and kidney function, blood lipids, and heart rate; and further promote the development of the disease. In addition, the patients were grouped based on the expressions of serum ADPN, hs-CRP, and sICAM-1 in the experimental group, and it was found that the incidence rate of cerebrovascular complications was 28%.

ADPN synthesized in adipose tissues possesses the antiatherosclerosis, anti-inflammatory, and insulin-sensitizing effects [25]. Lindstrom et al. reported that the level of serum ADPN is higher in patients with a longer course of disease (>10 years), which is caused by the deterioration of renal function with the prolongation of course [26]. In some studies, there is an association among cholesterol, duration of diabetes, age, and blood glucose control. Hs-CRP is a marker for coronary heart disease, and it is reported that hs-CRP is negatively correlated with the ADPN level in subcutaneous adipose tissues in patients with coronary heart disease. According to some studies, the level of sICAM-1 is higher in patients with cerebrovascular disease. During the 1-year follow-up after treatment, the total incidence rate of adverse cardiac events in the observation group is significantly lower than that in the control group, and the quality of life score is significantly higher than that in the control group [18]. The reason is that the incidence of cardiovascular events also increases with the increase of sICAM-1 level. Studies have confirmed that sICAM-1 is identified as a potent independent predictor for cardiovascular event and death, independent of most potential factors, especially other inflammatory markers including hs-CRP. In two prospective studies on patients with type 2 diabetes mellitus, the elevated level of plasma sICAM-1 is obviously associated with the increased risk of cardiovascular death, as well as renal function indexes [27]. Therefore, sICAM-1 is seemingly a marker for cerebrovascular complications. However, whether sICAM-1 has the biological activity associated with cardiovascular risk remains unclear. In this study, the content of ADPN in the experimental group was significantly reduced, while the content of hs-CRP and sICAM-1 was significantly increased. ADPN in the experimental group was negatively correlated with the incidence of cerebrovascular complications, while hs-CRP and sICAM-1 were positively correlated with the incidence rate of cerebrovascular complications. Activation of neuroglia worsens the pain, and neuroglia-based immunoinflammatory response plays an important role in cerebrovascular disease. Injecting glial cell line-derived neurotrophic factor (GDNF) can significantly reduce the expression of S100, indicating that the analgesic mechanism of GDNF is related to the inhibition on activation of astrocytes [28]. According to previous reports, the activation of astrocytes caused by cerebrovascular disease can be inhibited by GDNF through multiple pathways, in which GDNF can suppress the growth of afferent nerve fibers and the expression of neuropeptide Y that causes neuropathic pain [29]. This study found that the levels of S100 and NSE in the experimental group increased significantly, while the level of BNDF decreased significantly. Moreover, the cerebrovascular hemodynamic detection showed that the experimental group had evidently lower Vs, Vd, and Vm, and evidently higher PI, similar to previous studies [17]. The above research findings reveal that hs-CRP, sICAM-1, ADPN, and other indexes will be changed when cerebrovascular complications occur, which can provide theoretical support for predicting the development of disease.

In conclusion, a series of experiments in this study confirm that there are changes in the hepatic and renal function, blood lipids, and hemodynamics in patients with hypertensive cerebrovascular complications, further promoting the development of disease. Such effects can be further verified through animal experiments in the future. This study provides a theoretical basis for the pathogenesis, prevention, and treatment of hypertensive cerebrovascular complications, as well as new ideas for further research.

## Figures and Tables

**Figure 1:** Blood lipid indexes detected. In the experimental group, the content of TC, TG, and LDL obviously rises (*p* < 0.05), while the content of HDL obviously declines compared with those in the control group (*p* < 0.05). ^a^*p* < 0.05 vs. the control group.

**Table 1:** Clinical data of patients.

Parameter	Control group	Experimental group
Sample size	50	50
Number of males	26	25
Mean age (years old)	42 ± 11	43 ± 12
Mean weight (kg)	46 ± 10	48 ± 11
BMI (kg/m^2^)	20.9 ± 1.5	21.4 ± 1.2
Number of patients with grade 1 hypertension	15	17
Number of patients with grade 2 hypertension	20	21
Number of patients with grade 3 hypertension	15	12

**Table 2:** Serum hepatic and renal function indexes.

Group	AST (U/L)	ALT (U/L)	SCR (*μ*mol/L)	BUN (mmol/L)
Control group	22.4 ± 2.1	33.8 ± 2.4	50.7 ± 5.7	4.1 ± 1.2
Experimental group	88.8 ± 2.8^a^	78.7 ± 1.2^a^	113.9 ± 1.2^a^	15.3 ± 1.0^a^

Note: the content of AST, ALT, SCR, and BUN in the experimental group is significantly increased (*p* < 0.05). ^a^*p* < 0.05 vs. the control group.

**Table 3:** Blood pressure and heart rate.

Group	Systolic blood pressure (mmHg)	Diastolic blood pressure (mmHg)	Heart rate (beats/min)
Control group	85 ± 1.2	78 ± 0.9	70 ± 5
Experimental group	105 ± 1.5^a^	99 ± 1.2^a^	100 ± 3^a^

Note: the systolic and diastolic blood pressure and heart rate are all obviously increased in the experimental group compared with those in the control group (*p* < 0.05). ^a^*p* < 0.05 vs. the control group.

**Table 4:** Levels of serum ADPN, hs-CRP, and sICAM-1.

Group	ADPN (mg/L)	sICAM-1 (ng/mL)	Hs-CRP (mg/L)
Control group	12.5 ± 1.6	235.5 ± 50.4	2.4 ± 1.4
Experimental group	3.0 ± 0.8^a^	528.7 ± 61.4^a^	4.8 ± 1.0^a^

Note: in the experimental group, the content of ADPN is evidently decreased (*p* < 0.05), while that of hs-CRP and sICAM-1 is evidently increased. ^a^*p* < 0.05 vs. the control group.

**Table 5:** Content of serum S100, NSE, and BNDF.

Group	S100 (ng/L)	NSE (ng/L)	BNDF (ng/L)
Control group	0.85 ± 5.6	10.5 ± 5.4	4.4 ± 1.4
Experimental group	1.5 ± 3.8^a^	22.7 ± 6.4^a^	1.4 ± 1.0^a^

Note: in the experimental group, the levels of S100 and NSE are significantly increased (*p* < 0.05). ^a^*p* < 0.05 vs. the control group.

**Table 6:** Cerebrovascular complications.

Group based on indexes	Incidence rate of cerebrovascular complications
ADPN low-expression group	18%
ADPN high-expression group	10%
Hs-CRP low-expression group	12%
Hs-CRP high-expression group	16%
sICAM-1 low-expression group	10%
sICAM-1 high-expression group	18%

Note: there are 14 cases of postoperative complications in the experimental group, with an incidence rate of cerebrovascular complications of 28%.

**Table 7:** Cerebrovascular hemodynamic detection results.

Group	Vs (cm/s)	Vd (cm/s)	Vm (cm/s)	PI
Control group	88.5 ± 5.6	40.5 ± 5.4	46.4 ± 1.4	1.0 ± 0.2
Experimental group	83.5 ± 3.8^a^	28.7 ± 6.4^a^	25.4 ± 1.0^a^	1.5 ± 0.6^a^

Note: the experimental group has evidently lower Vs, Vd, and Vm (*p* < 0.05), and evidently higher PI (*p* < 0.05). ^a^*p* < 0.05 vs. the control group.

**Table 8:** Correlation of serum ADPN, hs-CRP, and sICAM-1 levels with incidence rate of hypertensive cerebrovascular complications.

Item	Incidence rate of hypertensive cerebrovascular complications	
	*r*	*p*
ADPN	-0.40	<0.05
Hs-CRP	+0.49	<0.01
sICAM-1	+0.45	<0.05

Note: in the experimental group, ADPN is negatively correlated with the incidence rate of cerebrovascular complications (*p* < 0.05), while hs-CRP and sICAM-1 are positively correlated with the incidence rate of cerebrovascular complications (*p* < 0.05).

## Data Availability

The datasets used and/or analyzed during the current study are available from the corresponding author on reasonable request.
